This article has been retracted.

# Single-Cell Transcriptomics Analysis of the Pathogenesis of Tendon Injury

**DOI:** 10.1155/2022/7887782

**Published:** 2022-09-13

**Authors:** Haibo Zhao, Ting Liang, Yijie Tang, Dongxu Zhu, Qian Lin, Jinli Chen, Jun Fei, Tengbo Yu, Yingze Zhang

**Affiliations:** ^1^Department of Sports Medicine, Affiliated Hospital of Qingdao University, Qingdao 266000, China; ^2^Department of Emergency, State Key Laboratory of Trauma, Burn and Combined Injury, Daping Hospital, Army Medical University, Chongqing 400042, China; ^3^Trauma and Emergency Center, The Third Hospital of Hebei Medical University, Shijiazhuang 050051, China

## Abstract

Tendon injury repair has been a clinical challenge, and little is known about tendon healing scar generation, repair, and regeneration mechanisms. To explore the cellular composition of tendon tissue and analyze cell populations and signaling pathways associated with tendon repair, in this paper, single-cell sequencing data was used for data mining and seven cell subsets were annotated in the tendon tissue, including fibroblasts, tenocytes, smooth muscle cells, endothelial cells, macrophages, T cells, and plasma cells. According to cell group interaction network analysis, pattern 4 composed of macrophages was an important communication pattern in tendon injury. Furthermore, the heterogeneity of M1 macrophages in tendons, the correlation of KEGG enriched pathway with inflammatory response, and the core regulatory role of the transcription factor NFKB and REL were observed; in addition, the heterogeneity of T cell isoforms in tendons was found and indicated that different isotypes of T cells involve in different roles of tendon injury and repair. This study demonstrated the heterogeneity of M1 macrophages and T cells in the tendon tissue, being involved in different physiological processes such as tendon injury and healing, providing new thinking insights and basis for subsequent clinical treatment of tendon injury.

## 1. Introduction

Tendon is a unique connective tissue with mechanical properties, which is capable of connecting muscles and bones, with the function of distributing, regulating, and transmitting the forces exerted by muscles on connecting structure, enabling the body to maintain posture or generate movement [1, 2]. This tendon connecting muscles and bone has a strong tear resistance and tensile strength and maintains a stable movement of the bone.

About 1/1,000 people develop tendon or ligament injury each year, and also, the incidence of tendon injury accounts for 46% of musculoskeletal injury [3]. Tendon injury is a common clinical disease, often accompanied by pain and impaired function, divided into acute tendon injury and chronic tendon injury, which can be caused by external cause (trauma) and internal cause (excessive tension) [4–6]. The damage repair process consists of three stages: wound healing, cell proliferation, and tissue remodeling. However, tendon healing is extremely slow and inefficient due to the lack of cellularity of the tendon tissue and growth factors, and the structural integrity and mechanical strength of the tendon are significantly inferior to the normal undamaged tendon [7–9]. Thus, the repair of tendon injury remains an immense challenge clinically, mainly due to the limited tendon healing capacity and our limited understanding of the underlying biology of tenocytes and the regulatory mechanisms of tendon injury occurrence [10].

The development of single-cell RNA sequencing (scRNA-Seq) technology combining single-cell isolation and RNA sequencing to enable analysis of the transcriptome at the single-cell level is an important tool for studying cellular heterogeneity and is changing many areas of biology [11]. scRNA-Seq technology is able to help identify different cell types and their expressed genes and to study cell heterogeneity and biological processes.

Tendon injury repair strategies have made many new directions and advances in recent years, currently mainly including gene therapy, stem cell therapy, platelet-rich plasma (PRP) therapy, growth factors, drug therapy, and tissue engineering [12]. In this paper, single-cell transcriptomes were drawn and analyzed by analyzing the cellular heterogeneity between healthy and tendon injury samples and by using single-cell transcriptomics. Studies at the single-cell level have explored the biological process of tendon injury involving each cell subpopulation, looking forward to providing some new ideas for therapeutic strategies for tendon injury.

## 2. Materials and Methods

### 2.1. Patient Information

This study was conducted according to the principles contained in the Declaration of Helsinki. Ethics was demonstrated by the Ethics Committee of the Affiliated Hospital of Qingdao University. All participants provided written informed consent for sample collection and subsequent analyses.

### 2.2. Reagents and Instruments

The trypan blue solution was purchased from Thermo Fisher Scientific. The erythrocyte lysate was obtained from Beyotime. The automated cell counter (Countess 3; Invitrogen) was obtained from Thermo Fisher Scientific.

### 2.3. Single-Cell Isolation

One of the straight head ophthalmic scissors and straight and elbow microtweezers each were one set of instruments, and two sets were prepared and placed in 50 mL flasks and soaked in 70% alcohol for 30 min. Tendon tissue was removed from the 4°C refrigerator, with a diameter not greater than 0.2~0.3 cm; placed on cell culture dishes; and gently washed three times with PBS buffer (no calcium and magnesium ions). Small pieces of tissue to approximately 1 mm^3^ were fragmented with straight head ophthalmic scissors; all described above were performed on ice boxes, adding 5 × tissue volumes of 3 mg/mL collagenase I and 3 mg/mL collagenase complex, and digested at 37 °C for 15 to 20 min. The 10 *μ*L cell suspension was placed in 10 *μ*L trypan blue solution and mixed with 10 *μ*L on the counting plate to observe the cell status and density of the incomplete and small; digestion was continued and detected every 30 min. After complete digestion, the enzyme digestion reaction was terminated with 10% serum, and a 40 *μ*m cell screen was filtered, and the cell suspension was collected. They were washed supplemented with 1 mL PBS buffer and centrifuged at 400 × g for 5 min. The supernatant was discarded, and 2 mL of erythrocyte lysate was added and reacted for 3 to 5 min. After the reaction, centrifuges were centrifuged at 400 × g at 5 min. The supernatant was discarded, and the cells were resuspended with 200 *μ*L of 1 PBS solution containing 0.04% BSA. 10 *μ*L cell suspension was placed in 10 *μ*L trypan blue solution and mixed, and 10 *μ*L was added to the cell count plate, and the total cell number and cell activity were detected by cell technology instrument.

### 2.4. Single-Cell Sorting

Samples were prepared into a single-cell suspension, requiring uniform cell size and cell mass and fragments < 5%, cell viability ≥ 85%, cell concentration, and total cells ≥ 1 × 10^6^ cell/mL. Cell labeling was performed based on the 10x Genomics Chromium™ system. The Gel Beads containing Barcode information is mixed with the cells, enzymes, and isolated oil beads to form GEMs (Gel Beads-In-Emulsion, meaning the oil droplets surrounding the cells and the enzyme mixture). Each gel bead was equipped with a large number of probes consisting of the Read1 sequence, a 16 bp 10x cell barcode (Barcode), a 10 bp UMI sequence (Unique molecular identifier, a unique molecular identifier), and a 30 bp Poly (dT). In each GEM, the mRNA released after cell rupture was reverse-transcribed into a cDNA with barcode. Then, the cDNA from all cells was collected together and amplified for sequencing library construction following the standard procedure of Illumina sequencing library construction.

### 2.5. Quality Control (QC) of Single-Cell Transcriptome Data with Sample Integration

The raw data from single-cell transcriptome sequencing were aligned by using the CellRanger (V1.1) software package from 10x Genomics and the RH38 reference genome. After obtaining the gene expression matrix by CellRanger, QC removed cells with mitochondrial gene ratio > 10% and 200 < number of genes < 5000. After filtering, a total of 93,621 cells were selected for subsequent analysis. Finally, the gene expression matrices of all samples were integrated by Seurat V.4 to eliminate batch effects between the different samples. Downstream analysis of the CellRanger matrices was performed using R (4.0.3) and the R package Seurat (4.0.0).

### 2.6. Dimension Reduction and Clustering

The filtered gene expression matrices were normalized by default parameters using the LogNormalize function in Seurat v.4. The top 2,000 variable genes were then identified using the “vst” method in the Seurat FindVariableFeatures function. Variables “nCount_RNA” and “percent.mito” were regressed out and PCA analyzed using the top 2,000 variable genes. UMAP was then performed on the top 50 major components to visualize the cells. Meanwhile, the PCA reduced data were cluster analyzed with Seurat v.4 with a resolution set to 1.0 to obtain a good clustering effect.

### 2.7. Reintegration of Macrophages and T Cells

Reintegration and aggregation of macrophages and T cells were performed using Seurat v.4. Specifically, the macrophages and T cells in all samples were reintegrated using the first 30 dimensions after the PCA (principal component analysis), and in the clustering step, the resolution parameters were set to 0.8 and 0.5, respectively, with 14 subclusters for macrophages and 10 subclusters for T cells.

### 2.8. Differential Gene Expression Analysis

Differential gene expression analysis was performed using the Findallmarkers functional function in Seurat V.4. For each cell cluster, it is compared to the other cells.

### 2.9. Gene Function Annotation

Because the clusterProfiler tool is characterized by supporting the statistical analysis and visual analysis of the functional profiles of gene and gene clusters, it was selected for the GO differential gene enrichment visualization analysis.

### 2.10. The CellChat Tool Analyzed the Interactions between the Various Cell Populations, as well as the Various Subpopulations of Macrophages and T Cells

To investigate cell to cell communication and differences between cells, we used iTALK (https://github.com/Coolgenome/iTALK) and CellChat (https://github.com/sqjin/CellChat) R package, which analyzed scRNA-Seq data. To determine cell-to-cell-to-cell communication, we analyzed the expression of ligands and receptors on cells using iTALK and thus inferred cellular communication. The average expression of the ligands and receptors needs to be greater than 0.01 to account for the communication between them. After obtaining the average expression levels of the ligands and receptors on the different cells using the iTALK software, the data were normalized using TBtools and the heat maps were generated. In addition, we used iTALK to analyze and visualize differences in cellular communication between different cell groups. The signaling pathway network was analyzed and visualized using the cell chat technology.

### 2.11. Statistical Analysis

All data analyses and visualization were conducted using R software (version 3.6, R Foundation for Statistical Computing, Austria).

## 3. Results

### 3.1. Single-Cell Transcriptome Sequencing Process and Single-Cell Gene Expression Profiles

Three healthy tendon samples and diseased tendon samples were performed for single-cell sequencing and data analysis according to map cellular gene expression profiles (Figure 1(a)). After quality control and filtration methods, 93,621 effective cells were obtained. UMAP cell clustering using unsupervised clustering of effective cells yielded a total of 24 different cell clusters (Figure 1(b)). Based to marker gene annotation of each cell cluster, seven cell populations containing fibroblasts, tenocytes, endothelial cells, smooth muscle cells, macrophages, plasma cells, and T cells were identified (Figure 1(c)). The distribution and expression level of marker gene in each cluster group were analyzed (Figures 1(d) and 1(e)). COL1A1 with high expression level in all seven cell populations and the most expression was found in tenocytes and smooth muscle cells. IL7R is mainly expressed in T cells, CD68 in macrophages, ACTA2 in smooth muscle cells, and CCL14 and SELE in endothelial cells, and MMP3 expression is higher in fibroblasts. The distribution of each cell cluster in the samples is shown in Figure 1(f). Heat map for the top 10 differential genes of each cluster is shown in Figure 1(g).

### 3.2. Cell Population Communication Analysis

Ligand-receptor circle maps were used to visualize the contribution of cell populations to ligand-receptor pairs. In Figure 2(a), tenocytes and fibroblasts are the main outputs of the whole cell population, regulating physiological homeostasis, tendon healing, tissue reconstruction, and other processes in the tendon tissue. Using cell chat to simulate cell-to-cell communication, cell chat divides cell communication into five patterns, as shown in Figure 2(b), where macrophages belong to a communication pattern 4. Analyzing heat map (Figure 2(b)), shock map (Figure 2(c), and bubble plot (Figure 2(d)), it is shown that the pathways are involved in TNF and CXCL and thus might participate in inflammatory response and cell migration at tendon injury.

### 3.3. KEGG Pathway Enrichment and Gene Set Variation Analysis (GSVA) of Macrophage Populations

Macrophages and B cells were further analyzed by UMAP, with a marked heterogeneity between tendon injury and healthy samples, and were increased markedly in tendon injury. The distribution of marker gene expression in the cell population is shown in Figures 3(c) and 3(e), significantly increasing the distribution of M1 macrophages in injured tendon tissues. The top 10 differential gene expressions are shown by a heat map, and KEGG pathway enrichment analysis was mainly enriched in IL-17 signaling and AGE-ARGE as well as TNF signaling (Figures 3(d), 3(f), and 3(g)).

GSVA is exhibited in Figure 4(a). This study evaluated whether different metabolic pathways were enriched by converting the expression matrix of genes from different samples to expression matrix of gene sets from different samples. The gene set variant score matrix was plotted based on the pathway enrichment results, and MAFG was enriched between M1 and M2 macrophages. The results of scenic analysis of macrophages and B cells in the tendon tissue in tendon injury and healthy samples showed that NFKB and REL expression is heterogeneous in tendons and plays an important role in the tendon injury and repair and healing stage (Figure 4(b)). Compared with type 2 macrophages, NFKB and REL are significantly regulated in M1 macrophages.

### 3.4. KEGG Pathway Enrichment and Cell Communication Analysis of T Cell Populations

The UMAP dot plot shows that T cells produced seven phenotypes in the tendon, as shown in Figure 5(a); except for RPS4Y1+T cell population, the other six phenotypes of T cells were significantly increased in tendon damaged tissue shown in Figure 5(b). PBX4+T, LUM+T, CXCL8+T, and CXCL 13+T, CD8+T were heterogeneous in tendons (Figures 5(c) and 5(d)). The GO enrichment analysis and the KEGG pathway analysis indicated that they were mainly involved in protein folding, a topologically incorrect protein response, and a cellular thermal response. Biological processes mostly occur in the extracellular matrix containing the organs. Protein processing in the endoplasmic reticulum and antigen presentation are the two pathways with the largest gene proportion in KEGG enrichment pathway (Figures 5(e) and 5(f)). Cell chat inferred the number of T cell subtype communication patterns, with LUM+T involved in pattern 2. To analyze the signaling pathway contribution, in pattern 2, mainly IGF, PARs, and CXCL pathways were involved in network interaction (Figures 5(g) and 5(h)). Impact maps and bubble maps of the T cell subpopulation and signaling pathway communication network are shown in Figures 5(i) and 5(j). The results showed that under the outgoing pattern, pattern 2 recognition revealed that the cell group LUM+T coordinated with the signaling pathways IGF, PARs, and CXCL that belonged to pattern 2 to send out signals.

## 4. Discussion

Tendon biology is key to understanding the mechanisms of tendon differentiation [13]. Studies of single-cell sequencing in the tendon tissue have been reported earlier, while groups other than the tendon cell population were rarely reported, which is not conducive to the in-depth study of the pathogenesis of tendon injury, healing, repair, etc. [14, 15]. Tendon repair is a tightly coordinated cellular cascade of events leading to the restoration of tendon continuity [16]. We used single-cell sequencing to build on basic tendon tissue grouping and differential gene expression analysis and also performed advanced data analysis to infer cell communication networks using newly developed gene expression software [17]. Based on the cell communication network, the inferred cell interaction pattern 4 involved in cell populations was further grouped, differential genes and transcription factors.

We classified and annotated subgroup single-cell sequencing data from healthy tendon tissue and annotated seven cell populations, respectively, fibroblasts, tenocytes, smooth muscle cells, endothelial cells, macrophages, and plasma cells. Mapping the expression of marker gene in the tendon tissue, each gene expression in different cell populations is specific, suggesting the rationality and reliability of cell sorting. For interaction communication network inference using CellChat, communication patterns were divided into five and interactions between the cell groups were involved in tendon healing and repair. Among them, pattern 4 mainly macrophages participates in the interaction, and pathway analysis found that the main pathways are TNF and CXCL, involved in inflammatory and immune responses, which is consistent with the results of inflammatory and immune responses of tendon injury in tendon tissue [18].

Further cellular annotation of macrophages identified M1 and M2 macrophages according to the marker gene annotation and increased the expression distribution of the proinflammatory factor producing M1 macrophages in tendon-damaged tissue, and correspondingly, M2 decreased, which is possibly involved in anti-inflammation and tissue tendon regeneration. In the analysis of the KEGG pathway, M1 macrophages were mainly enriched in the IL-17 signaling pathway and AGE-ARGE as well as TNF signaling, involved in inflammatory and immune responses. The results of transcription factor analysis showed that the heterogeneity of MAFG, NFKB, and REL in M1 and M2 had a significant regulation strength and played a core role in M1, laying the foundation for exploring tendon injury and repair and healing.

Finally, the isoform heterogeneity of T cells revealed seven isoforms of T cells, where PBX4+T, LUM+T, and CXCL8+T as well as CXCL 13+T and CD8+T were heterogeneous in tendon injury. In the analysis of interaction networks, pattern 2 where IGF, PARs, and CXCL pathways contribute highly affects tissue growth and development, promotes cell separation and value appreciation, and releases inflammatory mediators and cell migration.

## 5. Conclusion

We performed data mining for tendon injury and healthy tissue based on single-cell sequencing data, in addition to basal tendon tissue grouping and annotation, mainly analyzing macrophage and T cell population heterogeneity, and how they are involved in tendon injury and repair. Seven cell populations in tendon tissue, as well as the heterogeneity of M1 and M2 macrophages in tendon tissue, were proved, which are involved in different roles of tendon injury or repair; the KEGG pathway enrichment and transcription factors were analyzed, and the transcription factors NFKB and REL have strong regulatory strength in cells. Analysis of T cell populations revealed that the apparent heterogeneity of some isoforms is extremely involved in different roles in tendon repair.

## Figures and Tables

**Figure 1:** Tendon tissue cell gene map. (a) The 10x Genomics scRNA-Seq process of healthy and diseased tendon tissue samples. (b) UMAP dimensionality reduction clustering based on the gene matrix. Each cluster contains cells from both healthy and disease samples. (c) Marker gene defines cell taxa and performs cell annotation. Each cell population contains cells from both healthy and disease samples. (d) Expression of the selected marker gene in each cell cluster. Point size indicates the number of gene expressed cells, and shades of color indicate gene expression levels. (e) Representative marker genes mapping on the UMAP map. Color gradient indicates the level of gene expression. (f) The proportion of cells in cell clusters in each sample. 0, 1, 3, 14, and 16: fibroblasts; 2, 4, 5, 9, 10, and 13: tendon cells; 7, 11, 20, 21, and 23: endothelial cells; 6, 8, 17, 18, and 19: smooth muscle cells; 12: macrophages; 22: plasma cells; 15: T cells. (g) Heat map of top 10 gene expressions in each cluster of cells. Yellow is upregulated, and purple is downregulation of gene expression levels.

**Figure 2:** Cell population communication network. (a) Circle map of each cell group of the tendon tissue. The size of the outer circle color indicates the number of cells, cells emitting arrows indicate ligands, and arrows pointing to cells indicate receptors. (b) Global communication patterns and main signals of cell group. Color transition from blue to yellow indicates greater cell populations or major signal contribution. (c, d) Outgoing communication pattern recognition of secretory cells. (c) River plot. (d) Dot plot. The bubble size indicates the signal contribution.

**Figure 3:** Analysis of the macrophages and B cell populations. (a, b) Annotation analysis of specific macrophages and the B cell group. (a) The subset annotation in health and disease tendon cells. (b) left: the subset annotation in healthy tendon cells; right: the subset annotation in disease tendon cells. (c) The maker gene distribution in cell clusters. (d) The heat map of top 10 differential gene expressions of each cluster in macrophages and the B cell group. (e) The distribution of macrophages and the B cell group in the sample. (f) M1 macrophages and (g) M2 macrophage KEGG pathway analysis.

**Figure 4:** Heat map of the variant score matrix of gene sets. (a) Heat map of the transcription factor enrichment score matrix based on the KEGG pathway annotation. (b) Heat map of the regulator activity of each cell (SCENIC analysis).

**Figure 5:** A subpopulation analysis of T cell populations. (a) UMAP analysis of T cell group subsets. (b) UMAP plot of T cell population of healthy and diseased tendon tissue samples. Left: T cell subpopulation in healthy tendon cells; right: T cell subpopulation in disease tendon cells. (c) Marker gene expression and distribution in the T cell subgroup. (d) Distribution of T cell subgroup in samples. (e) The GO enrichment analysis. (f) KEGG pathway enrichment analysis. (g) T cell subgroup ligand-receptor interaction network diagram. The size of the outer circle color indicates the number of cells; the cells emitting the arrow indicate the ligand and the cells pointing to the receptor. (h) The global communication pattern and the main signal between the subgroups. Color transition from blue to yellow indicates greater cell populations or major signal contribution. (i, j) Outgoing communication pattern recognition of secreted cells. (i) River plot. (j) Dot plot. The bubble size indicates the signal contribution.

## Data Availability

The datasets used or analyzed during the current study are available from the corresponding authors on reasonable request.
